# Study on the Clinical Value of Noninvasive Prenatal Testing in Screening the Chromosomal Abnormalities of the Fetus in the Elderly Pregnant Women

This article has been retracted.

**DOI:** 10.1155/2022/2977128

**Published:** 2022-09-28

**Authors:** Zhiping Gu, Mengmeng Du, Tianhui Xu, Chunyan Jin

**Affiliations:** Department of Medical Genetics and Prenatal Diagnosis, Taizhou People's Hospital, Taizhou, 225300 Jiangsu, China

## Abstract

**Introduction:**

To explore the clinical value of noninvasive prenatal testing (NIPT) in screening the chromosomal abnormalities of the fetus in the elderly pregnant women.

**Materials and Methods:**

Between January 2020 and December 2021, 1949 elderly pregnant women underwent NIPT in our hospital. At the same time, 236 elderly pregnant women received invasive prenatal diagnosis, and the pregnancy outcomes were followed-up.

**Results:**

When NIPT was used for prenatal screening of fetal chromosomal aneuploidy, its diagnostic coincidence rate for trisomy 21 was the highest, with a coincidence rate of 90.00%, and the diagnostic coincidence rate for other chromosomal abnormalities was the lowest, only 22.22%. The sensitivity, specificity, positive predictive rate, and negative predictive rate for T21 by NIPT were 100%, 99.97%, 94.28%, and 100%; for T18 were 100%, 99.92%, 72.22%, and 100%, respectively; and for T13 were 100%, 99.95%, 50%, and 100%, respectively. Patients with high risks according to NIPT results further received invasive prenatal diagnosis, and 18 cases were excluded from the follow-up. For the remaining 1933 cases in the NIPT group, there was an incidence of 2.28% of adverse pregnancy outcomes. For the remaining 234 cases in the Amniocentesis group, there was an incidence of 1.28% of adverse pregnancy outcomes. There was no significant difference between the two groups (*P* > 0.05). The diagnostic rate of fetal chromosomal abnormalities in pregnant women under 40 years old was about 0.39-0.79%; however, the risk for people over 40 is relatively high at 1.32-4.44%.

**Conclusion:**

The noninvasive prenatal screening of fetal DNA in the second trimester of pregnancy for elderly pregnant women has high application value in the prediction of pregnancy outcome. The high risk of pregnancy can be determined by detecting trisomy 21, 18, and 13 syndromes, and the probability of adverse pregnancy outcome increases.

## 1. Introduction

With the continuous development and progress of society, great changes have taken place in people's ideas. The number of late marriage and late childbirth groups is increasing. In addition, the country has fully opened the second and third child policy, which has led to an increase in the number of elderly pregnant women in China, showing an upward trend [1]. The risk of pregnancy and delivery of older pregnant women is relatively high. The probability of adverse pregnancy outcomes is relatively high. Abortion, stillbirth, and fetal malformation account for a large proportion. For example, trisomy 21, 18, and 13 syndromes are common fetal chromosomal abnormalities. The fetus is prone to physical structure deformity or nerve damage after delivery, which has a great impact on the newborn family and economic burden [2]. Therefore, it is very necessary to do a good job in the screening of fetal malformations and chromosomal abnormalities in the second trimester of pregnancy for older pregnant women. It can accurately screen fetal malformations, which is of great significance for the prediction of adverse pregnancy [3]. At present, the gold standard to screen fetal chromosomal abnormalities in clinical practice is invasive prenatal diagnosis, that is, amniocentesis diagnosis [4]. However, this diagnostic method is traumatic, and will increase the probability of abortion in elderly pregnant women. At the same time, it has the risk of amniotic fluid infection. The diagnostic application has certain limitations [5]. In recent years, many studies have shown [6–8] that there is a certain amount of free fetal DNA in the peripheral blood of pregnant women in the second trimester of pregnancy, so the noninvasive screening of fetal DNA in the second trimester of pregnancy was born. Noninvasive prenatal testing (NIPT) has been reported to have high sensitivity and specificity for detecting common chromosomal aneuploidies (trisomies 21, 18, and 13), with low false positive and false negative rates [9]. Moreover, clinical experiments have indicated that NIPT has a good detection effect in both high-risk and low-risk populations of serological screening, and the detection efficiency is much higher than that of serological screening [10]. In some cases, it can replace amniocentesis, and the detection rate and diagnostic coincidence rate of fetal chromosomal abnormalities are higher.

In this study, we investigated the clinical value of NIPT in screening the chromosomal abnormalities of the fetus in the elderly pregnant women.

## 2. Materials and Methods

### 2.1. General Clinical Data

A total of 1949 elderly pregnant women who received NIPT in our hospital from January 2020 to December 2021 were enrolled in this study. According to the informed consent and NIPT results, 236 elderly pregnant women directly received amniotic fluid prenatal diagnosis at the same time, and the pregnancy outcomes were followed-up. The expected age of the study subjects was between 35 and 50 years old, and the average age of pregnant women was 39.48 ± 3.83 years old. The gestational weeks of NIPT ranged from 12 to 28 weeks, with an average of 16.18 ± 1.05 weeks.

Inclusion criteria: (1) the elderly pregnant women refer to the pregnant women whose actual age is ≥35 at the expected delivery date; (2) all pregnant women included in the study were required to complete pregnancy outcome follow-up.

Exclusion criteria: (1) pregnant women with previous history of induced labor or delivery of fetus with abnormal chromosome, or pregnant women with history of unexplained abortion, stillbirth, abnormal fetus, and neonatal death; (2) pregnant women with definite chromosomal abnormalities or who have given birth to children with monogenic genetic diseases or genetic metabolic diseases; (3) pregnant women who have given birth to children with congenital heart disease, open spina bifida, anencephaly, and other abnormalities; (4) having a family genetic history or having a history of marriage between close relatives within three generations; (5) pregnant women who had suffered from severe infectious diseases in the early stage of pregnancy; (6) fetal ultrasound showed multiple soft index abnormalities; (7) gestational weeks <12 weeks or >22 weeks; (8) pregnant women with malignant tumors; (9) receiving allogeneic blood transfusion, transplantation surgery, allogeneic cell therapy, and so on within one year; (10) other conditions that the physician felt significantly affected the accuracy of the results.

### 2.2. Methods

For pregnant women who meet the inclusion and exclusion criteria, amniotic fluid prenatal diagnosis is recommended when the NIPT indicated the positive results of chromosomal abnormalities. According to the principle of statistics, the detection rate of fetal chromosomal aneuploidy between NIPT and amniocentesis groups was counted.

### 2.3. NIPT Detection

The pregnant women have signed informed consent before NIPT testing. 5 ml of maternal peripheral blood samples were selected and temporarily stored in a refrigerator at 4°C. Samples will be excluded if hemolyzed or stored for more than 8 hours before plasma separation. Blood specimens were processed as follows: centrifugation at 4°C, 1600 g for 10 min, and plasma was carefully collected and distributed into 2.0 ml Eppendorf tubes. The plasma was centrifuged again at 16000 g at 4°C for another 10 min. The upper layer of plasma was carefully divided into 2.0 ml new Eppendorf tubes, each containing approximately 600 ml of plasma, stored in a refrigerator at -80°C. Repeated freezing and thawing of plasma should be avoided before the experiment. DNA extraction, library construction, and sequencing were performed using Nucleic Acid Extraction Kit (BGI, Shenzhen, China) on BGIseq-500 sequencing platform (BGI). Fetal chromosome aneuploidies (T21, T18, and T13) detection kit (Combinatorial Probe-Anchor Synthesis Sequencing Method) (BGI) was used for library construction. Sequencing was performed using Universal Reaction Kit for Sequencing (Combinatorial Probe-Anchor Synthesis Sequencing Method) (BGI). Z-score set the range of -3 and 3 as the threshold to evaluate the risk of chromosomal aneuploidies. *Z* = 3 was considered as the cut-off value, and the sample was classified as high-risk of chromosomal abnormalities when ∣ *Z*  | >3, *Z* between -3 and 3 represented the sample was classified as low risk [11].

### 2.4. Amniotic Fluid Puncture Test

The amniocentesis procedure was as follows: Pregnant women with indications should have B-ultrasound first to determine the placenta position and fetal condition, so as to avoid accidental injury to the placenta. If there is no B-mode ultrasound, palpation can be used to find the part of the floating fetal body with large cystic sex and easy to touch, and the placenta can also be avoided. After selecting the needle entry point, the skin was disinfected, disinfection towel was spread, local anesthesia was given, and the waist needle with the needle center was used to pierce the selected point vertically; when the needle passed through the abdominal wall and uterine wall, it was disinfected twice, and the needle core was removed. 2 ml of amniotic fluid was aspirated with a 2 ml syringe and discarded. This section of amniotic fluid may contain maternal cells. Then, 20 ml of amniotic fluid was aspirated with a 20 ml empty needle, which was placed in two disinfection tubes and capped. Take out the needle, cover with sterilized gauze, compress for 2-3 minutes, and the pregnant woman stayed in bed for 2 hours. The amniotic fluid was centrifuged for 5-10 minutes, the above clear liquid was used for biochemical test, and the sediment was used for cell culture or DNA extraction. Amniotic fluid cells were cultured in a 5% carbon dioxide incubator at 37°C. When the results of NIPT indicated that trisomy 21, 18, and 13 were at high risk or indicative of abnormal chromosome number, G-banding chromosome karyotype analysis + chromosome microarray analysis (CMA) were performed in amniotic fluid cell culture; If NIPT results suspect that there may be other chromosomal abnormalities or gene level microdeletions and microduplications, amniotic fluid cell culture G-banding chromosome karyotype analysis + gene chip detection shall be given to make a definite diagnosis.

### 2.5. Follow-Up

The pregnancy outcomes of all pregnant women were followed-up, except those with abnormal results in prenatal diagnosis and induced labor including outpatient, telephone, and Internet follow-ups.

Follow-up contents: (1) Pregnant women who have low-risk NIPT results or who refuse to undergo prenatal diagnosis despite high-risk NIPT results should follow-up, whether there are structural or soft index abnormalities in B-ultrasound results after NIPT. (2) Whether peripheral blood chromosome examination is performed after delivery, or whether induced labor tissue microarray is performed for induced labor. (3) Whether the appearance of induced labor fetus or newborn is normal. (4) Whether the weight of the newborn is normal. (5) At the same time, it is judged according to whether the newborn's appearance and physical and intellectual development are abnormal. The follow-up was completed in 2-6 months after termination of pregnancy.

### 2.6. Statistical Analysis

SPSS (version 22.0) software was used for statistical processing of all data in this study. The sensitivity, specificity, and positive predictive rate of NIPT were evaluated. The coincidence between the chromosome aneuploidy in NIPT and prenatal diagnosis of amniotic fluid was compared. Chi-square test was used to analyze data conforming to normal distribution. The difference was statistically significant when *P* < 0.05.

## 3. Results

### 3.1. Test Results of Each Group

A total of 1949 subjects were included in the study. The number of positive women who underwent NIPT test was 42, and the positive rate was 2.15%. Further amniotic fluid puncture test identified 10 cases of T21, 4 cases of T18, 0 case of T13, 7 cases of sex chromosome aneuploidy, 9 cases of other chromosome aneuploidy, and 12 cases of chromosome copy number variation. In the amniocentesis group, 236 cases of elderly pregnant women directly received amniotic fluid puncture test. The results confirmed 9 cases of T21, 1 case of T18, 3 cases of sex chromosome abnormality, 2 cases of other chromosome aneuploidy, and 3 cases of chromosome copy number variation. The positive cases were 18, and the positive rate was 0.92%. When NIPT was used for prenatal screening of fetal chromosomal aneuploidy, its diagnostic coincidence rate for trisomy 21 was the highest (90.00%), and the diagnostic coincidence rate for other chromosomal aneuploidy was the lowest (22.22%), as shown in Table 1.

### 3.2. Invasive Diagnosis Results for CNV

Among the 236 cases that received amniotic fluid puncture test, the results indicated that there was 1 pathogenic case and 1 likely pathogenic case, as shown in Table 2.

### 3.3. Pregnancy Outcome Follow-Up

According to the prenatal diagnosis results, 16 pregnant women in the NIPT group and 2 pregnant women in the amniocentesis group chose to induce labor, and these participants were excluded from our follow-up. For the remaining 1933 cases in the NIPT group, the follow-up results showed that there were 35 abortions, 3 stillbirth, and 6 fetal malformations, a total of 44 adverse pregnancy outcomes with an incidence of 2.28%. For the remaining 234 cases in the amniocentesis group, there were 2 abortions, 0 stillbirth, and 1 fetal malformations with 1.28% adverse pregnancy outcomes. There was no significant difference between the two groups, *P* > 0.05, as shown in Table 3.

### 3.4. Screening Efficiency of NIPT for Common Fetal Chromosomal Aneuploidy and Other Chromosomal Abnormalities

The sensitivity, specificity, positive predictive rate, and negative predictive rate of trisomy 21 screened by NIPT were 100%, 99.97%, 94.28%, and 100%, respectively. The sensitivity, specificity, positive predictive rate, and negative predictive rate of trisomy 18 were 100%, 99.92%, 72.22%, and 100%, respectively, and the sensitivity, specificity, positive predictive rate, and negative predictive rate of trisomy 13 were 100%, 99.95%, 50%, and 100%, respectively, as shown in Table 4.

### 3.5. Relationship between Maternal Age and Fetal Chromosome Abnormality

A total of 1949 elderly pregnancies were included in this study and underwent NIPT. Among them, 42 cases received amniotic fluid prenatal diagnosis after NIPT test was positive, and 236 cases directly received invasive prenatal diagnosis. The results of fetal chromosomal abnormalities are listed in the following table according to the age of pregnant women, and the true positive rate of fetal chromosomal aneuploidy at all ages is calculated, as shown in Table 5. The diagnostic rate of fetal chromosomal abnormalities in pregnant women under 40 years old was about 0.39-0.79%; however, the risk for people over 40 is relatively high at 1.32-4.44%.

## 4. Discussion

Birth defects are one of the common diseases of newborns in China, and chromosomal abnormalities are one of the important causes of birth defects [12]. Among them, autosomal abnormalities can be manifested in different degrees of mental retardation, growth retardation, appearance, and organ deformity, and sex chromosome abnormalities can be manifested in gonadal hypoplasia, hermaphroditism, etc. At present, there is no effective treatment for these chromosomal abnormalities. We can only try to avoid the birth of such children through secondary prevention, especially children with trisomy 21 syndrome.

NIPT is a new noninvasive detection method. It uses a new generation of high-throughput sequencing technology to sequence fetal free DNA fragments in maternal peripheral blood, and then judge whether the fetus has abnormal chromosome aneuploidy. Ben et al. and Smid et al. had confirmed that cell-free fetal DNA (cffDNA) existed in the peripheral blood of pregnant women, and its metabolic law met the requirements of prenatal screening [13, 14], but the technology at that time could not achieve high-throughput detection. With the rapid development of high-throughput detection technology, NIPT was gradually used in clinical detection [15, 16]. At present, the superiority of NIPT technology has been widely recognized at home and abroad. Many clinical pilots have conducted large-scale data research on NIPT and found that the positive predictive value of NIPT for T21 is as high as 80~89%, and the positive predictive value of T18 is also greater than 60%, both of which are significantly higher than the positive predictive value of routine serological screening (T21 is 3.4%~4.2%, T18 is 8.3%). Moreover, the missed screening rates of T21 and T18 detected by NIPT were 0.3% and 0.2%, respectively, which were significantly lower than those of serological screening (3.6%~5.2% for T21 and 0.6% for T18) [17]. It can be seen that NIPT has absolute advantages over the traditional serological prenatal screening in the screening of T21 and T18. In addition, it has the characteristics of noninvasive operation, which effectively solves some problems existing in interventional prenatal diagnosis, and even in some aspects, it can replace prenatal diagnosis. It has been widely concerned by all walks of life and has gradually become a research hotspot [18].

Prenatal examination and prenatal diagnosis are the main measures used to eliminate fetal deformities and prevent birth defects. The traditional serological screening is mainly aimed at the common chromosomal diseases of the fetus (T21, T18). Although early screening can be carried out, the detection rate is low and the false positive rate is high. Even if the prenatal screening results of pregnant women are high-risk, there is only a 5% chance that the fetus can be diagnosed with chromosomal diseases [19]. The high risk of screening results will increase the mental and psychological burden of pregnant women and their families to a certain extent, and the low-positive detection rate makes many people feel lucky and give up prenatal diagnosis, which leads to the loss of the original significance of prenatal screening and the birth of children. In fact, this kind of missing screen occurs almost every year, causing lifelong regret. Conventional prenatal diagnosis methods (such as chorionic puncture, amniocentesis, amniotic fluid, umbilical vein puncture) require uterine puncture of pregnant women, which is traumatic and has the risk of fetal loss and infection. As a result, a considerable number of pregnant women are afraid of this method, so their compliance is reduced. In addition, whether the soft index of systematic ultrasound is abnormal or not, is often used to evaluate the risk that the fetus may be associated with chromosomal diseases [20]. However, due to the nonspecificity of these soft indices, their sensitivity is not high. Limited by this, ultrasound doctors must have many years of experience in prenatal diagnosis before they can find these abnormalities. However, there are certain differences in the current medical level in China, which limits its application to a certain extent [21].

The existing norms of prenatal screening and prenatal diagnosis in China require that pregnant women with serological screening results at critical risk can undergo NIPT, while older pregnant women with high-risk results or expected childbirth age ≥35 years old are still recommended to choose interventional prenatal diagnosis as the first choice [22]. However, with the continuous deterioration of the living environment and the increasing number of planned pregnancies, especially older pregnancies, after the liberalization of the two child policy, the proportion of high-risk and older pregnant women has doubled. However, the poor compliance caused by the fear of trauma of prenatal diagnosis among pregnant women and the shortage of medical resources have brought enormous pressure to prenatal diagnosis [23]. Therefore, this study intended to actively find a more optimized screening program in order to reduce the missed screening rate, reduce the number of cases requiring interventional prenatal diagnosis, and achieve the purpose of reducing the operation risk as much as possible.

In this study, 1949 pregnant women with high risk of prenatal screening or advanced age (NIPT group) required NIPT first. The results of NIPT showed high risk in 42 cases which received further invasive prenatal diagnosis, the results of NIPT were low-risk in 1907 cases, and no missed screening was found at present according to the pregnancy outcome. At the same time, 236 pregnant women received invasive prenatal diagnosis for further confirmation.

The elderly pregnant women included in the study first had NIPT, and then had further prenatal diagnosis when NIPT results were at high risk. Compared with the elderly pregnant women who had direct interventional prenatal diagnosis, there was a coincidence rate of 42.8% in fetal chromosomal abnormalities between the two methods. Similarly, according to Table 2, there was no significant difference between NPT test results and invasive test results of copy number variants (CNVs). CNVs are ubiquitous in the human genome, and CNVs-related diseases, including Digeorge syndrome (22Q11), CRIP-Du-Chat syndrome (5P-), and 1P36 deletion syndrome, have been documented [24]. Moreover, there is increasing evidence that CNV is associated with adverse pregnancy outcomes [25]. In our study, there is no significant difference in the detection rate of fetal chromosomal abnormalities between the screening of high-risk pregnant women and the direct interventional prenatal diagnosis. Therefore, we infer that if some elderly pregnant women refuse to directly carry out interventional prenatal diagnosis, they can be asked to choose NIPT first. If NIPT results are high-risk, then carry out interventional prenatal diagnosis, which should be equivalent to the detection rate of direct interventional prenatal diagnosis. At least, the probability of missing fetal chromosomal aneuploidy is very small. This approach can reduce a large part of the operation risk and also provide an alternative and relatively reliable way for pregnant women with surgical contraindications. Relieve the mental pressure of pregnant women and their families, improve compliance, reduce the risk of surgery, and reduce the work intensity of prenatal diagnosis practitioners. At present, the cost of NIPT is relatively high, which hinders its further promotion in clinical practice. Of course, as the government pays more attention to this cause and the cost of high-throughput sequencing is further reduced, this problem is expected to be solved. The wide application of NIPT is just around the corner. In addition, according to the data in Table 5, the diagnostic rate of fetal chromosomal abnormalities in pregnant women under the age of 40 was lower than 1%; however, the risk for people over 40 was relatively high, could be up to 4.44%. In order to prevent missed screening and reduce the chance of puncture surgery, different prenatal screening and prenatal diagnosis schemes can be adopted for elderly pregnant women in stages.

It should be noted that during the follow-up, a very small number of pregnant women were informed of the high risk of NIPT and directly terminated their pregnancy without further prenatal diagnosis. Therefore, normal fetuses may be abandoned. This should be related to the pregnant women's insufficient understanding of the false positive of NIPT, leading to the wrong choice. In fact, at present, the diagnostic coincidence rate of NIPT for T21was the highest (90.00%), which was significantly higher than that of other groups (see Table 1). Therefore, NIPT can only be used as a high-precision screening and cannot replace prenatal diagnosis to detect all chromosomal abnormalities. There are still false positives. To the best of our knowledge, NIPT is a noninvasive prenatal screening technique for fetal aneuploidies. NIPS is based on high-throughput sequencing to detect cffDNA in maternal blood [26]. Therefore, the most likely reason for false positives is that fetal and fetal cffDNA accounts for insufficient proportion of total cffDNA. Therefore, pregnant women with positive NIPT results must undergo interventional prenatal diagnosis to determine whether the fetus has chromosome or gene-level abnormalities. With our in-depth study of NIPT, we hope that more pregnant women can correctly understand the relationship between NIPT and interventional prenatal diagnosis and make correct and scientific choices. This can also promote the benign and sustainable development of NIPT.

There are some shortcomings of this study. Firstly, there were some undiagnosed cases in the high-risk groups tested by NIPT. Moreover, because of the low incidence of trisomy 18 and trisomy 13, age-stratified studies could not be performed as in trisomy 21. Therefore, more studies with larger sample sizes are expected to be carried out in the future to provide more data support for optimizing prenatal screening and diagnosis strategies for elderly pregnant women.

In conclusion, the noninvasive prenatal screening of fetal DNA in the second trimester of pregnancy for older pregnant women has a high application value in the prediction of pregnancy outcomes. The high risk of pregnancy can be determined by detecting trisomy 21, 18, and 13, and the probability of adverse pregnancy outcomes increases. Therefore, noninvasive prenatal screening of fetal DNA in the second trimester of pregnancy should be popularized in clinical practice, so as to reduce the probability of adverse pregnancy outcomes in older pregnant women.

## Figures and Tables

**Table 1:** Test results of each group.

Groups	T21	T18	T13	Sex chromosome aneuploidy	Other chromosome aneuploidy	Chromosome copy number variation	Total cases	Positive rate (%)
NIPT group	10	4	0	7	9	12	42	2.15%
Amniocentesis group	9	1	0	3	2	3	18	0.92%
Coincidence rate (%)	90.00	25.00	—	42.86	22.22	25	42.86	42.8%

**Table 2:** Invasive diagnosis results for CNV.

Maternal age	Gestational age	NPIT site	Invasive diagnosis	Pathogenesity
38	16	del 16p13.11-p12.3^b^	del 16p13.12-p12.3^b^	Pathogenic
42	17	Dup 22q11.21	Dup 22q11.21	Likely pathogenic

**Table 3:** Follow-up of pregnancy outcomes in patients with different risks.

Groups	*N*	Abortion	Stillbirth	Fetal malformation	Incidence of defects
NIPT group	1933	35	3	6	2.28%
Amniocentesis group	234	2	0	1	1.28%
*χ* ^2^		0.9724			
*P*		0.3241			

**Table 4:** Efficiency of NIPT in screening common fetal chromosomal aneuploidy and other chromosomal abnormalities.

	Sensitivity	Specificity	Positive predictive value	Negative predictive value
21-trisomy syndrome	100%	99.97%	94.28%	100%
18-trisomy syndrome	100%	99.92%	72.22%	100%
13-trisomy syndrome	100%	99.95%	50.00%	100%

**Table 5:** Analysis of chromosome screening in pregnant women of different age groups.

Age (years)		35	36	37	38	39	40	41	42	43	≧44	Total
N		782	257	262	183	126	98	76	68	52	45	1949
Diagnosis of chromosome abnormality	T21	2	1	0	1	1	1	1	1	0	1	9
	T18	0	0	1	0	0	0	0	0	0	0	1
	T13	0	0	0	0	0	0	0	0	0	0	0
	Sex chromosome abnormality	1	0	0	0	0	1	0	0	1	0	3
	Other exceptions	1	0	1	0	0	0	0	1	1	1	5
	Total	4	1	2	1	1	2	1	2	2	2	18
True positive rate (%)		0.51	0.39	0.76	0.54	0.79	2.04	1.32	2.94	3.85	4.44	0.92

## Data Availability

Data appears in the submitted article.
